RETRACTED

# Polyvinylpyrrolidone K-30-Based Crosslinked Fast Swelling Nanogels: An Impeccable Approach for Drug's Solubility Improvement

**DOI:** 10.1155/2022/5883239

**Published:** 2022-08-26

**Authors:** Muhammad Usman Minhas, Kifayat Ullah Khan, Muhammad Sarfraz, Syed Faisal Badshah, Abubakar Munir, Kashif Barkat, Abdul Basit, Mosab Arafat

**Affiliations:** ^1^College of Pharmacy, University of Sargodha, Sargodha City Punjab, Pakistan; ^2^Quaid-e-Azam College of Pharmacy, Sahiwal, Punjab, Pakistan; ^3^College of Pharmacy, Al Ain University, Al Ain Campus, Al Ain, UAE; ^4^Faculty of Pharmacy, University of Lahore, Punjab, Pakistan; ^5^Faculty of Pharmacy, Superior University Lahore, Punjab, Pakistan

## Abstract

Poor solubility is a global issue of copious pharmaceutical industries as large number of drugs in development stage as well as already marketed products are poorly soluble which results in low dissolution and ultimately dosage increase. Current study is aimed at developing a polyvinylpyrrolidone- (PVP-K30-) based nanogel delivery system for solubility enhancement of poorly soluble drug olanzapine (OLP), as solubilization enhancement is the most noteworthy application of nanosystems. Crosslinking polymerization with subsequent condensation technique was used for the synthesis of nanogels, a highly responsive polymeric networks in drug's solubility. Developed nanogels were characterized by percent entrapment efficiency, sol-gel, percent swelling, percent drug loaded content (%DLC), percent porosity, stability, solubility, in vitro dissolution studies, FTIR, XRD, and SEM analysis. Furthermore, cytotoxicity study was conducted on rabbits to check the biocompatibility of the system. Particle size of nanogels was found with 178.99 ± 15.32 nm, and in vitro dissolution study exhibited that drug release properties were considerably enhanced as compared to the marketed formulation OLANZIA. The solubility studies indicated that solubility of OLP was noticeably improved up to 36.7-fold in phosphate buffer of pH 6.8. In vivo cytotoxicity study indicated that prepared PVP-K30-based formulation was biocompatible. On the basis of results obtained, the developed PVP-K30-co-poly (AMPS) nanogel delivery system is expected to be safe, effective, and cost-effective for solubility improvement of poorly soluble drugs.

## 1. Introduction

Poor solubility is a major issue of sundry pharmaceutical industries as about 40% of already marketed drugs and about 75-90% drug candidates in development stage are poorly aqueous soluble [1] calling for exploring effective strategies to improve their solubility and dissolution so as to enhance their efficacies for desirable therapeutic responses [2–4]. These drug products leaves gastrointestinal tract (G.I.T) before the dissolution and originate inadequate ADME properties leading to reduced clinical effects and dosage escalation [5, 6]. Various strategies have been investigated for solubility enhancement such as polymeric composites [7], polymeric nanoparticles [8], polymeric microneedles [9], polymeric microbeads [10], cocrystals [11], solid lipid nanoparticles (SLNs) [12], micelles [13], hydrogels [14], amorphous solid dispersions [12], liposome [15], nanosuspension [16], nanoemulsion, nanoplex [17], self-emulsifying drug delivery system (SEDDS), inclusion complexation with cyclodextrins, dendrimers, and nanocapsule [18–20].

RETRACTED

Among the aforementioned strategies, due to high swelling ability, high drug loading and entrapment efficiency, stability, reduced particle size, and biocompatibility, nanogels have gained enormous interest in designing the nanocarrier system for solubilization enhancement of poorly soluble drugs [21–24]. Nanogels are solvent swollen nanosized soft polymeric networks that have the ability of absorbing and retaining large amount of water with being dissolved [20, 23, 25]. They are nanoscale hydrogels holding the abilities of hydrogels as well as nanocarriers [20]. They are highly crosslinked networks capable of hosting both hydrophilic and hydrophobic drugs [26, 27]. They are soft nanosized (20-200 nm) and innovative nanocarrier system that could play a dynamic role in addressing various issues faced in pharmaceutical industries related to new chemical entities (NCEs) and marketed products such as inadequate dissolution, poor aqueous solubility, stability, and bioavailability [28–30].

In the current study, olanzapine (OLP) is used as a model drug. It is one of the most appropriate 2^nd^ generation atypical antipsychotic drug approved by US FDA as first line therapy for the treatment of psychotic disorders schizophrenia, anxiety, depression, and acute mania with bipolar disorder [31–34]. OLP binds and antagonizes many receptors (serotonin, dopamine, histamine, and alpha-1 adrenergic receptors) [35, 36]. Even though olanzapine (OLP) is a poorly soluble drug (0.0942 mg/mL) which is an impediment to the schizophrenia treatment and leads to poor absorption and unreliable pharmacokinetic profile [37, 38], for this purpose, in the current study, we developed the nanogel drug delivery system to improve the solubility and bioavailability profile of olanzapine.

For polymeric nanocarriers, water loving polymers and monomers offering the most auspicious solution [39]. Hydrophilic polymers/monomers have been widely used for solubility improvement of poorly soluble drugs. Hydrophilic (water loving) polymers shows maximum hydration (90%) as compared to hydrophobic polymers [40]. Previously, our research group has developed poloxamer-407, poly ethylene glycol-4000, and *β*-cyclodextrin-based nanogels and nanomatrices, respectively [41–43]. Keeping in view, in the current study, polymer polyvinylpyrrolidone (PVP-K30) is investigated for the synthesis of nanogels in which seven (7) different formulations have been developed by changing the ratio of the polymer, monomer, and crosslinker as compared to our previously reported nanogel formulations. PVP-K30 is a water loving nontoxic synthetic polymer with excellent absorbency and biocompatibility [44, 45]. Many researchers reported PVP-K30 in different delivery systems to enhance the solubility of poorly soluble drugs [46, 47].

RETRACTED

## 2. Materials and Methods

### 2.1. Chemicals

The active pharmaceutical ingredient (API) of OLP (MW = 312.4 g/mol) was achieved from the Global Pharm. PK. Initiator ammonium persulfate (APS) (MW = 228.18 g/mol), polymer polyvinylpyrrolidone PVP-K30 (MW = ~40000 g/mol), and monomer (AMPS) (MW = 207.24 g/mol) were purchased from Sigma-Aldrich.

### 2.2. Methods

#### 2.2.1. Synthesis of Polyvinylpyrrolidone- (PVP-K30-) Based Nanogels

Polyvinylpyrrolidone- (PVP-K30-) based chemically crosslinked nanogels were prepared with some amendments in our previously published polymerization technique [42, 48]. Initially, mixture of polymer polyvinylpyrrolidone and monomer 2-acrylamido-2-methylpropane sulfonic acid (AMPS) was prepared in distilled water using hotplate magnetic stirrer at 300 rpm. The accurately weight amount of crosslinking agent methylene bis-acrylamide (MBA) was solubilized separately in distilled water (20 mL) and ethanol (10 mL) mixture (2 : 1). After this, weight amount (2 percent with respect to monomer) of reaction initiator APS was added into the PVP/AMPS mixture. Finally, the PVP/AMPS/APS mixture was added into already prepared solution of MBA with continuous stirring (300 rpm) at 50°C, and then the whole mixture was poured into round bottom flask. A round bottom flask was immediately fitted with condenser followed by the reflux-condensation process at 75-85°C. Finally, the prepared gel was sieved and placed in oven for the purpose of drying. The proposed schematic diagram and feed ratio of ingredients used in PVP-K30-based nanogels are shown in Figure 1 and Table 1, respectively.

#### 2.2.2. Drug Loading of Naive Nanogels

Developed PVP-K30-based nanogels were loaded with OLP by using the previously reported swelling diffusion method [43]. For drug loading, initially two percent OLP solution (weight/volume) was prepared with methanol and distilled water mixture at the ratio of 4 : 1. After this, on to the drug solution, specific quantify of developed nanogels was added and sonicated for specific time (30-40 minutes). OLP/nanogel mixture was kept for 24 hours at room temperature for swelling and loading purpose which was then lyophilized (for 4-5 hours) and characterized by various parameters.

RETRACTED

## 3. In Vitro Characterization of Nanogels

### 3.1. Structural Analysis

Fourier transform infrared spectroscopy (FTIR) was carried out for structural analysis and to confirm any interactions between drug and ingredients. FTIR (ATR-FTIR, Tensor-27 series, Bruker Co. DEU) was carried out at resolution of 4 cm^−1^ for pure drug olanzapine (OLP), polymer polyvinylpyrrolidone (PVP-K30), monomer AMPS, and OLP-loaded nanogels formulation. Scanning range for all samples were kept from 4000 to 600 cm^−1^.

### 3.2. Particle Size Analysis

Particle size of the delivery system is an important factor in solubility and bioavailability enhancement of hydrophobic drugs. For this purpose, a homogenous suspension of prepared optimized nanogels was determined for particle size using particle size analyzer (Malvern instrument, United Kingdom). Prepared nanogel samples were analyzed in ultrapure water filtered with membrane filter having a pore size of 0.22 *μ*m [49].

### 3.3. Surface Morphology Using SEM

Surface morphology of prepared PVP-K30-based formulations was examined by using scanning electron microscope (JSM5910, Japan) with high resolution. For this purpose, PVP-K30-based nanogel samples were spotted on double-adhesive tape attached to gold plated aluminum stub.

### 3.4. Powder X-Ray Diffraction Analysis

Samples of pure drug olanzapine (OLP) and optimized nanogel (loaded & blank) formulations were subjected to X-ray diffraction studies to determine the degree of crystallinity of OLP after loading into the nanogels using X-ray Diffractometer (JDX3522, Japan) as crystallinity is closely related to solubility. PXRD data was recorded in range of 0-60° at 2-theta.

## 4. In Vitro Studies of Prepared Nanogels

### 4.1. Swelling Analysis

Swelling behavior was carried out to analyze the swelling capacity of the prepared nanogels. For this purpose, accurately measured quantity of naive nanogels was placed in unfilled tea bags and then suspended in specified labeled containers of corresponding solutions of pH 6.8 and 1.2 at normal temperature of 37°C ± 0.5. Nanogel samples were taken out at predetermined time intervals, i.e., 02, 05, 10, 15, 20, 30, 40, 50, 60, 90, 120, and 150 minutes followed by blotted with filter paper. The samples were weighed and returned to their respective containers. Equation (1) was used to calculate swelling index [50].

(1) $$\begin{array}{c} Q\;\left(\text{swelling index}\right)=\frac{W_{2}}{W_{1}}, \end{array}$$

where *W*_2_ indicates the weight of swollen, and *W*_1_ indicates weight of dried nanogel sample.

RETRACTED

### 4.2. Sol-Gel Studies

Sol-gel studies were carried out to analyze the percentage of reactants converted into the product, i.e., to analyze the % crosslinked as well as uncrosslinked quantity of polymer (PVP-K30) and monomer (AMPS) in the nanogel structure. Sol-gel analysis was done using Soxhlet extraction technique. Accurately measured nanogels, i.e., 500 mg (W1) were taken and subjected to Soxhlet extraction process for approximately 4-5 hours. After extraction process, samples were placed in oven till drying at 40°C and weighed again W2 in order to measure the % sol-gel fraction by applying Equations (2) and (3).

(2) $$\begin{array}{c} \text{Sol fraction }\left(\%\right)=\frac{\left(W_{1}–W_{2}\right)}{W_{1}}\times 100, \end{array}$$

(3) $$\begin{array}{c} \text{Gel fraction }\left(\%\right)=100-\text{Sol fraction}. \end{array}$$

*W*_1_ indicates the initial weight (dry) of nanogels, whereas *W*_2_ indicates the weight (dry) after extraction.

### 4.3. Entrapment Efficiency and Drug-Loaded Content

The entrapment efficiency (%) and drug loaded content (%) of PVP-K30-based nanogels were calculated by the absorption and extraction technique [51]. Specific quantity of OLP loaded nanogel formulations (100 mg) was dispersed in the specific solution (50 mL) of phosphate buffer of pH 6.8 followed by stirring at 100 rpm for 1 hour at room temperature. After this, the resultant suspension was filtered through membrane filter having the pore size of 0.45 *μ*m. The resultant solution was then analyzed using UV-spectrophotometer at *λ*-max 228 nm. %DLC and EE were calculated using Equations (4) and (5), respectively.

(4) $$\begin{array}{c} \%\text{DLC}=\frac{\text{Entrapped drug in formulation}}{\text{Weight of formulation}}\times 100, \end{array}$$

(5) $$\begin{array}{c} \%\text{EE}=\frac{\text{Actual drug contents in formulation}}{\text{Theoretical drug contents in formulation}}\times 100. \end{array}$$

### 4.4. Solubility Studies

Solubility studies were carried out to analyze the solubility of OLP enhanced by the developed PVP-K30-based nanogels. Solubility of OLP was studied at different pH conditions, i.e., pH 6.8 and pH 1.2 (phosphate buffer solution and HCl solution, respectively) as well as in distilled water. For this purpose, pure drug (OLP) and PVP-K30 nanogel formulations (100 mg) were dispersed in 20 mL of DW, phosphate buffer, and HCl solution separately with continuous stirring at 200 rpm for 24 hours. The solutions were then analyzed using UV-spectrophotometer at *λ*-max 228 nm [52].

RETRACTED

### 4.5. Stability and Porosity (%) Evaluation of Nanogels

ICH guidelines were followed to carry out the stability studies of OLP-loaded PVP-K30 nanogels [53]. For this purpose, formulations were placed in glass vials and kept at 40 ± 02°C with 75 ± 5% RH in the stability chamber. Various parameters such as any physical changes in the sample, % DLC, FTIR, and solubility efficiency were analyzed over the specific time period, i.e., six months.

Developed nanogels are highly porous structure which assists in the absorption and drug release from the system. % porosity of PVP-K30-based nanogels were found out using the solvent replacement method. Specific quantity of developed nanogels were weighted and suspended in water and weighted again followed by careful blotting and calculating of weight variation. The percent porosity of formulations was measured using Equation (6).

(6) $$\begin{array}{c} \text{Porosity }\left(\%\right)=\frac{\left(\text{Wh}-\text{Wd}\right)}{\rho V}\times 100. \end{array}$$

Wh represents the weight of saturated nanogels, Wd represents weight of dried nanogels, *ρ* indicates the density of DW, and V indicates the volume of formulation.

### 4.6. In Vitro Drug Release Studies

Drug release studies of prepared nanogel formulations (PNG1-PNG7) and reference product of olanzapine (OLANZIA) were performed in calibrated 6-station dissolution test apparatus (Curio-Pak.). Samples were placed in 500 mL of phosphate buffer (pH 6.8) and HCl solution (pH 1.2) at 50 rpm (37°C ± 0.5°C). Samples were placed in dissolution apparatus using the reported tea bag method. At predefined time intervals, samples were withdrawn (five mL) using a pipette and then diluted with equal volume of respective medium to keep the volume constant, and then the amount of drug release was quantified using spectrophotometer at ʎ-max 228 nm.

### 4.7. In Vivo Toxicity Evaluation

PVP-K30-based developed nanogel formulations are intended to administer orally; for this purpose, compatibility profile of nanogels with the biological environment was analyzed using the rabbit model. Toxicity study was conducted for 14 days in which test animals (rabbits) were randomly divided in to 2 groups, i.e., group C (controlled) and group T (treated) and then kept in cleaned cages. Naive nanogel formulations (5 g/kg) were given orally to group T, and then all animals were observed for water and food consumption, any irritation (ocular/skin), urination, salivation, tremors, general response behavior, diarrhea, mortality, etc. On the day 15^th^, blood samples were taken followed by slaughtering the animals of both groups for evaluation of blood biochemistry, hematological, liver profile, and weight variation of vital organs [54, 55].

RETRACTED

## 5. Results and Discussions

### 5.1. Particle Size Analysis

Large surface area and reduced particle size favor the process of disintegration, dissolution rate, absorption, and ultimately the bioavailability. Solubility of the poorly soluble drugs significantly enhanced when the particle size reduces and vice versa [56]. Nanosystem, i.e., nanogels/nanomatrices/nanosponges/nanoparticles are important and interesting platforms to enhance the solubility, dissolution rate, and bioavailability of poorly soluble drug entities. For particle size analysis, zeta sizer (Nano Zeta Sizer, United Kingdom) was employed. Single peak was observed which indicated that 81% of particle size of PVP-K30-based nanogels were 178.99 ± 15.32 nm as shown in Figure 2. Polydispersity index (PDI) was found 0.51 which indicates that nanogels have very low affinity of forming clusters. Nanotechnology greatly influences the biopharmaceutical performance of the system according to Noyes-Whitney equation, and reduced particle size leads to large surface area which in turn enhances solubility, dissolution rate, and bioavailability [57].

### 5.2. Fourier Transform Infrared Spectroscopy (FTIR)

The FTIR spectra of pure drug olanzapine (OLP), monomer 2-acrylamido-2-methylpropane sulfonic acid (AMPS), polymer polyvinylpyrrolidone (PVP-K30), and OLP loaded formulation (PNG-7) were recorded to confirm and analyze crosslinking between polymer and monomer as well as check any possible interaction between drug and excipients. FTIR spectra of all reactants have been presented in Figures 3(a)–3(d). The FTIR spectrum of pure AMPS was recorded that showed characteristic band at 1,658.59 cm^−1^ which was attributed to carbon and oxygen stretching (C=O). Principal peaks at 1,233.92 cm^−1^ and 1,371.74 cm^−1^ indicated the symmetrical stretching of sulfur and oxygen group (S=O) that indicated the existence of SO_3_H group in AMPS as shown in Figure 3(a). Strong absorption bands at 1,092.83 cm^−1^ and 941.96 cm^−1^ were recorded that represent the S-O-C group. Peak at 2,910.81 cm^−1^ suggested C-H stretching of the -CH_2_ group. FTIR spectrum of polymer PVP-K30 has shown characteristic peak at 1643.92 cm^−1^ which corresponds to amide C=O bond. Absorption band at 3441.43 cm^−1^ is attributed to O-H stretching of absorbed water (H_2_O) molecules while absorption peaks at 2886.11 cm^−1^ and 1415.24 cm^−1^ attributed to the C-H bonds, and peaks at 1260 cm^−1^ and 882 cm^−1^ are allocated to C-N stretching and breathing vibration of the pyrrolidone ring present in the PVP-K30 polymer, respectively, as shown in Figure 3(b) [58]. In the FTIR spectrum of pure drug olanzapine (OLP), characteristic peaks were observed at 3,265 cm^−1^ which was attributed to the N-H & O-H stretching, 1,593 cm^−1^ due to C=C, 2,960 cm^−1^ due to C-H, 1,391 cm^−1^ due to C=N, and 755 cm^−1^ due to C-S stretching as shown in Figure 3(c). FTIR band of OLP-loaded nanogels has shown that all the characteristic peaks of drug, polymer polyvinylpyrrolidone (PVP-K30), and AMPS were there with insignificant modifications as shown in Figure 3(d), which indicated the successful crosslinking of reactants and entrapment of drug OLP into the amorphous system of PVP-K30-based nanogels.

RETRACTED

### 5.3. Scanning Electron Microscopy (SEM)

In order to examine the surface morphology of the developed PVP-K30-based nanogel formulations, scanning electron microscopy was carried out at different magnifications using scanning electron microscope (JSM-6490A, Tokyo, Japan). SEM images were shown (Figure 4) that developed nanogels were highly porous and spongy. Numerous pores present in PVP-k30-based formulations can be ascribed to the presence of hydrophilic and ionic groups of polymer (PVP-K30) and monomer (AMPS). Upon contact with aqueous media, the porosity favors the nanogels for entrance and release of water and drug, respectively.

### 5.4. XRD Analysis

Figures 5(a)–5(c) present the X-ray diffraction (XRD) patterns of OLP, blank, and OLP-loaded formulation (PNG-7), respectively. The study was conducted for the purpose to evaluate the degree of crystallinity of pure OLP as well as to find out any possible alterations made in OLP nanocrystals after integrating it into the nanogel amorphous network. It is well known that crystalline drugs have poor aqueous solubility than amorphous form. According to the literature, solubility can be enhanced up to sixteen hundred times due to the amorphous form [59, 60].

The XRD pattern of pure olanzapine (OLP) displayed various characteristics peaks at diffraction angle of 2-theta (10-30°) which pointed of high crystalline nature of OLP as displayed in Figure 5(a). X-ray diffraction spectrum of unloaded PVP-K30 formulation displayed that there was lack of any significant peak which clearly indicated that the crystallinity of OLP by the amorphous nanogels has been effectively masked. In the XRD band of OLP-loaded formulation, the characteristics intense peaks of OLP were there (Figure 5(c)) but with distinct decrease intensity as compared to pure OLP. The broader peaks of OLP with noticeably decrease intensity indicated the successful incorporation of OLP in the amorphous nanogel network which may contributed in the rapid dissolution and solubility enhancement.

RETRACTED

### 5.5. Swelling Behavior of Nanogels

Swelling of the system has a huge and direct influence on drug release characteristics; that is why swelling properties of the developed polyvinylpyrrolidone- (PVP-K30-) based nanogel formulations were investigated [61]. Swelling study was carried out in both acid (1.2) and basic (6.8) pH medium to analyze the effect of pH medium as well as polymer PVP-K30, monomer (2-acrylamido 2-methyl propane sulfonic acid), and crosslinking agent MBA concentration on swelling. It was observed from the results that maximum swelling occurred in 2-10 minutes at both pH conditions (1.2 and 6.8), which was ascribed to the highly hydrophilic nature of PVP-K30 and AMPS [62]; moreover, nanogels are small size spongy materials that impart higher swelling abilities which in turn favor the abrupt drug release in aqueous medium [30]. All nanogel formulations have shown excellent swelling results at both higher and lower pH conditions but slightly more at basic pH (6.8) quantitatively as compared to acidic pH (1.2) as shown in Figures 6(a) and 6(b). This was due to the sulfonate anions (-SO_3_^−^) present in monomer (AMPS) and was protonated into -SO_3_H, due to the stout interaction between sulfonate groups resulted additional crosslinking that cause decreased swelling dynamics in acidic medium while in case of higher pH due to the strong electrostatic repulsion between -SO_3_^−^ groups as a result of ionization of some sulfonate ions triggered increased swelling dynamics [63, 64].

During swelling experiment, the effect of PVP-K30, AMPS, and crosslinking agent MBA concentration in nanogels was also analyzed. With increase in MBA concentration, swelling index was increased (PNG-6 and PNG-7) due to high crosslinking points in the system. According to Flory's theory, excessive crosslinking causes generation of additional crosslinking points during polymerization process which result in enhanced gelling network and swelling index [65]. The hydrophilic groups (-OH) of polymer (PVP-K30) and monomer (AMPS) and –NH groups introduced by the MBA during radical polymerization are responsible for favorable polymeric network-solvent interaction triggering solvent uptake [66]. Slight decrease was observed in swelling index with increasing mass ratio (Table 1) of polymer/monomer to MBA (PNG1-PNG5) that was due to the availability of less crosslinking points in the solution produced during free radical polymerization which resulted in inadequate gelling structure as shown in Figures 6(a) and 6(b).

### 5.6. Sol-Gel Analysis

Figure 7 has shown the sol-gel analysis of the prepared nanogels (PNG1-PNG-7). Sol-gel experiment was conducted in order to find out the uncrosslinked fraction of polymer (PVP-K30) and monomer (AMPS) in the nanogel structure. The results have shown good gelling fraction in all nanogel formulations. Sol fraction is the uncrosslinked components of the gel structure which was removed by extraction process. From sol-gel experiment, it was observed that gel fraction was gradually decreased, and sol fraction increased with increase concentration of polymer polyvinylpyrrolidone (PVP-K30) and monomer AMPS (PNG-1 to PNG-5). Decreased gelling fraction with increase polymer and monomer concentration may be due to excess of free radicals (active sites) produced during polymerization reaction in the system remained uncrosslinked due to less %wt of crosslinking agent (MBA). The ratio of all ingredients is shown in Table 1. Crosslinker is a key factor and directly related to gelling. The result showed that gelling fraction was significantly increased with increase in MBA concentration (PNG-6 and PNG-7) as shown in Figure 7. This may be attributed to the availability of more crosslinking point in the system, and maximum active site of polymer and monomer was crosslinked to form good gelling network.

RETRACTED

### 5.7. Solubility Studies

To determine the solubility of the pure drug OLP by developed PVP-K30-based nanogel formulations (PNG1-PNG7), surplus quantity of pure drug olanzapine (OLP) and nanogel formulations was dispersed in specific amount of DW, HCl, and phosphate solutions of pH 1.2 and 6.8, respectively, by using magnetic hotplate at 300 rpm at 37°C for 24 hrs. UV-spectrophotometer was used to analyze the absorbance both filtered solutions at wavelength of 228 nm.  Figure 8 presents the comparison of solubility of pure OLP and OLP-loaded nanogels, in DW, pH 1.2, and pH 6.8 buffer solutions. The solubility of OLP by developed nanogel formulations (PNG-1 to PNG-7) in DW was enhanced up to 33.39, 33.41, 32.01, 32.95, 29.11, 34.19, and 35.21 times, respectively. Similarly, the solubility of OLP by developed nanogel formulations (PNG-1 to PNG-7) in phosphate was improved by 34.51, 33.32, 32.23, 31.94, 29.99, 34.83, and 36.71 times, respectively, while the solubility was enhanced by nanogels in HCl buffer of pH 1.2 up to 33.99, 32.97, 31.88, 32.16, 31.29, 34.73, and 36.39 times, respectively, as compared to the solubility of pure OLP in distilled water, phosphate buffer of pH 6.8, and HCl buffer of pH 1.2.

Substantial enhancement in the solubility of the poorly soluble drug olanzapine may be attributed to the smaller particle size and larger surface area of the PVP-k3-based nanogels, wettability, and solubilizing effect of hydrophilic excipients (polyvinylpyrrolidone-K30 and AMPS) used and amorphous structure of nanogels which also confirmed by XRD analysis. Incorporation of poorly soluble drugs into hydrophilic polymeric matrix leads to enhanced solubility [67].

RETRACTED

### 5.8. Stability and Porosity (%) Analysis of Nanogels

Table 2 presents the data of porosity (%) of developed PVP-k30-based nanogels (PNG-1 to PNG-7). It was noted that the number of pores in the nanogel structure decreased by increasing the concentration of polymer polyvinylpyrrolidone-K30 (PNG-1 to PNG-3) and monomer AMPS (PNG-4 and PNG-5). This was may be due to the high feed content ratio of polymer PVP-K30 in PNG-2 and 3 with respect to the crosslinker MBA, due to which some concentration of polymer molecules remained uncrosslinked due to insufficient crosslinker. The observations did not match with the results of our previously reported studies in which the porosity was increased with the increase in polymer and monomer concentration [43]. In the current study, the feed content ratio of PVP-K30 and AMPS was higher as compared to the previously reported studies which indicated that the feed content ratio of all the ingredients such as polymer, monomer, and crosslinker is a crucial factor that affect the porosity, swelling, and sol-gel fraction as well as drug release. The average number of pores increased with the increasing of the concentration of crosslinking agent MBA (PNG-6 & PNG-7). This may be due to the high crosslinking points in the system due to MBA concentration, i.e., maximum portion of the polymer and monomer was crosslinked, and proper gel structure was formed which results in increased gel fraction as well as porosity as presented in Table 2.

Table 3 shows the data observed during the stability studies. The prescribed study of OLP-loaded PVP-K30-based nanogels over the specified time period, i.e., six months displayed that developed nanogels remained stable. No evident alteration/modification was noticed in physical texture, percent drug-loaded content values, FTIR spectrum, and solubility enhancement efficiency which overall endorsed the stability of the developed PVP-K30-based nanogel formulation.

### 5.9. In Vitro Dissolution Studies and Percent Drug-Loaded Content

To find out the in vitro drug OLP-release profile from polyvinylpyrrolidone- (PVP-K30-) based nanogel carrier system, dissolution study was performed in phosphate and HCl solutions of pH 6.8 and 1.2, respectively. Dissolution experiment was carried out for all prepared nanogel formulations (PNG1-PNG7) as well as for marketed product of olanzapine (OLANZIA) so that to compare the drug release with prepared nanogels. Quick and rapid drug release was observed in 5 to 10 minutes from all prepared nanogel formulations at both pH (1.2 and 6.8) but insignificantly more in 6.8 quantitatively as presented in Figures 9(a) and 9(b). Excellent and rapid drug release was attributed to the hydrophilic and highly amorphous nature of nanogels which favored high swelling and rapid drug release. Moreover, incorporation of a hydrophobic drug entity in a hydrophilic and amorphous polymeric network might result in its enhanced solubility as well as fast dissolution in the aqueous media because when water loving polymer/monomer dissolves, the entrapped drug presents itself as very fine particles for fast dissolution as illustrated in Figure 9(c).

RETRACTED

Quantitatively more and rapid OLP release in phosphate buffer was due to the sulfonate anions (-SO_3_^−^) present in monomer (AMPS) that were protonated into –SO_3_H, due to the stout interaction between sulfonate groups resulted more crosslinking which in turn cause decreased swelling ratio in acidic solution (1.2) while in case of basic pH due to the strong electrostatic repulsion between –SO_3_^−^ groups as a result of ionization of some sulfonate ions triggered increased swelling ratio and in turn, higher drug release was examined in higher pH 6.8 [61, 63].

Besides the effect of pH on dissolution rate and drug release characteristics, effect of polyvinylpyrrolidone-K30 (polymer), AMPS (monomer), and crosslinking agent concentration was also analyzed. In the first three formulations (PNG1-PNG3), polymer PVP-K30 was gradually increased while kept the concentration of remaining ingredients constant as presented in Table 1. It was observed that drug released was slightly decreased as shown in Figure 9. Similar results were observed in case of AMPS (monomer). This was due to less crosslinking points in the system because the crosslinking agent concentration was remained constant. Similarly, DLC and EE were also decreased with increasing polymer/monomer concentration as shown in Table 1. In formulations PNG-6 and PNG-7, the concentration of MBA was gradually increased while kept the polymer and monomer concentration constant. There was an observed increase in drug release as well as drug-loaded content as shown Figure 9. This was due to the more crosslinking points in the solution, and all active sites of polymer and monomer produced by the initiator were crosslinked to form good gelling structure.

In order to compare the developed PVP-K30-based nanogels, in vitro dissolution study was also carried out for commercially available OLP tablets (OLANZIA) in both pH conditions (6.8 and 1.2). It was observed that in comparison with the prepared nanogels, equal concentration of drug (OLP) was released in 40-60 minutes from the reference product in basic medium (pH 6.8) and 30-40 minutes in acidic medium as displayed in Figures 9(a) and 9(b). This significant difference with the reference product indicates that the solubility and drug release characteristics are significantly enhanced by the developed nanogels.

RETRACTED

### 5.10. In Vivo Toxicity Evaluation

As the developed nanogel drug delivery system intended to be administered orally, for this purpose, toxicity study was conducted to analyze the compatibility profile of the system. Toxicity study was performed in accordance with the United Kingdom Animals (Scientific Procedure) act, 1986, and associated guidelines. The procedure followed by the study was reviewed and approved by the Pharmacy Animal Ethics Committee, Department of Pharmaceutics, Faculty of Pharmacy, IUB-Pakistan. During the study, animals were carefully observed physically for water and food consumption, any irritation (ocular/skin), urination, salivation, tremors, general response behavior, body weight, diarrhea, mortality, etc. All the aforementioned physical parameters (Table 4) indicated that there no drastic change was observed.

After the 14^th^ day, all animals were slaughtered for the hematological biochemical examination in order to determine the effect of developed nanogels on the biological system. Blood samples from animals were immediately collected in EDTA tubes to avoid blood coagulation. The laboratory findings of hematological/biochemical tests were found normal which confirmed that prepared nanogels were safe and biocompatible as shown in Tables 5 and 6. Previously, similar observations are reported by Minhas et al. [50].

During toxicity study, the effect on weight of vital organs was also evaluated; for this purpose, vital organs of the animals (group C and group T) were carefully removed and immersed in formalin solution. No perceptible change was recorded in organ weights of both groups as presented in Table 7. So, conclusively, toxicity study indicated that the developed nanogels are biocompatible with the biological system.

## 6. Conclusion

To date, 70-90% drugs under development and about 40% marketed drugs are poorly soluble which greatly affect their pharmacokinetic profile. To tackle this common problem, in the current research, PVP-K30-based nanogels have been successfully prepared by free radical polymerization technique. XRD analysis indicated highly amorphous nature of nanogels which was the key factor in solubilization enhancement according to literature solubility that can be enhanced up to 1600 times by applying amorphous form. Solubility studies revealed that olanzapine (OLP) solubility is enhanced 36.7-fold by prepared nanogels. In vitro dissolution studies exhibited significantly higher and rapid release of OLP at both pH conditions (6.8 and 1.2) as compared with OLANZIA (reference product). Cytotoxicity evaluation endorsed the safely of nanogels. Conclusively, it could be mentioned that amorphous, spongy, and porous structure of the developed PVP-K30-based nanogels could made them an excellent choice for the solubility enhancement of poorly soluble drugs.

RETRACTED

## Figures and Tables

**Figure 1:** Proposed scheme of prepared PVP-K30-based nanogels.

**Figure 2:** Particle size measurement of prepared PVP-K30-based nanogels.

**Figure 3:** FTIR spectra of (a) monomer AMPS, (b) PVP-K30, (c) pure OLP, and (d) OLP-loaded formulation (PNG-7).

**Figure 4:** SEM micrographs of developed PVP-K30-based formulation (PNG-7) at different resolutions.

**Figure 5:** PXRD analysis of (a) drug olanzapine (pure), (b) blank nanogels, and (c) OLP-loaded nanogels (PNG-7).

**Figure 6:** (a) Swelling index of developed nanogels (PNG1-PNG7) at phosphate buffer of pH 6.8. (b) Swelling index of developed nanogels (PNG1-PNG7) at HCL buffer of pH 1.2.

**Figure 7:** Sol-gel analysis of developed nanogel formulations (PNG-1 to PNG-7).

**Figure 8:** Solubility of OLP in prepared nanogels (PNG-1 to PNG-7) and in DW, HCl, and phosphate solutions of pH 6.8 and 1.2, respectively.

**Figure 9:** (a) Dissolution profile of prepared PVP-K30-based formulations and RP OLANZIA in phosphate buffer of pH 6.8. (b) Dissolution profile of prepared PVP-K30-based formulations (PNG1-PNG7) and RP OLANZIA in HCl solution (pH 1.2). (c) Mechanism illustrating the drug release from the prepared PVP-K30-based formulations.

**Table 1:** The ratio of PVP-K30 (g), AMPS (g), methylene bisacrylamide (MBA) (g), and percent drug-loaded content (%DLC) in nanogels.

S/N	Formulation code	PVP-K30	AMPS	MBA	%DLC^∗^
01	PNG-1	01	04	0.5	85.86 ± 1.21
02	PNG-2	02	04	0.5	84.05 ± 2.01
03	PNG-3	03	04	0.5	80.14 ± 2.06
04	PNG-4	03	06	0.5	78.71 ± 1.99
05	PNG-5	03	08	0.5	68.06 ± 2.04
06	PNG-6	03	04	01	90.04 ± 1.78
07	PNG-7	03	04	02	92.89 ± 2.00

^∗^Values are measured as mean ± SD (*n* = 3).

**Table 2:** % porosity of PVP-k30-based nanogels (PNG-1 to PNG-7).

Sr. no.	Formulations	Excipients/reactants	Porosity^∗^ (%)
01	PNG-1	PVP-k30 (polymer)	82.054 ± 1.124
02	PNG-2		78.982 ± 1.046
03	PNG-3		75.846 ± 1.476
04	PNG-4	AMPS (monomer)	76.438 ± 1.354
05	PNG-5		74.854 ± 0.995
06	PNG-6	MBA (crosslinker)	85.681 ± 2.001
07	PNG-7		89.246 ± 1.763

^∗^Values measured as mean ± SD (*n* = 3).

**Table 3:** Findings of stability studies of OLP-loaded nanogels.

Sr. no.	Parameters	Fresh reading	After 3 months	After 6 months
1	FTIR analysis	Carried out	Not changed	Not changed
2	%DLC	92.89 ± 2.00	92.001 ± 1.89	91.997 ± 2.013
3	Physical texture	Yellowish appearance	Not changed	Not changed
4	Solubility improvement of OLP by nanogels	Improved up to 36.7-fold	Prominent change not observed	Prominent change not observed

RETRACTED

**Table 4:** Physical observations examined during toxicity study in both groups.

Parameters observed	Group C	Group T
1. Body weight (kg)		
Prior treatment	01.86 ± 0.14	01.86 ± 0.16
7^th^ day	01.88 ± 0.15	01.87 ± 0.15
14^th^ day	01.89 ± 0.13	01.86 ± 0.14
2. Food consumption (g)		74.01
Prior treatment	71.56 ± 2.12	72.65 ± 2.99
7^th^ day	73.02 ± 2.32	74.34 ± 2.08
14^th^ day	72.87 ± 2.83	74.01±2.56
3. Water consumption (mL)		
Prior treatment	190.04 ± 2.00	188.87 ± 2.79
7^th^ day	191.46 ± 2.85	191.63 ± 2.66
14^th^ day	193.10 ± 2.45	191.09±3.02
4. Dermal toxicity	Not observed	Not observed
5. Ocular toxicity	Not observed	Not observed
6. Mortality rate	No	No

Values are measured as mean ± SD (*n* = 3).

**Table 5:** Hematological examination of animals of both groups.

Laboratory findings	Group C	Group T
RBC count (10^6^/mm^3^)	05.69 ± 1.02	05.82 ± 1.07
WBC count (10^9^/L)	06.12 ± 0.45	06.17 ± 0.73
Platelet count (10^9^/L)	209.11 ± 2.21	204 ± 2.69
Neutrophils (%)	56.62 ± 1.95	53.76 ± 1.53
Monocytes (%)	03.78 ± 0.23	03.84 ± 0.06
Eosinophil (%)	03.33 ± 0.34	03.68 ± 0.29
Hemoglobin (g/dL)	13.13 ± 0.36	13.25 ± 0.44
Lymphocytes (%)	40.25 ± 1.13	41.16 ± 1.00

Values are measured as mean ± SD (*n* = 3).

**Table 6:** Biochemical examination of liver profile of group C and group T.

Biochemical analysis	Group C	Group T
Cholesterol level (mg.dL^−1^)	62.45 ± 2.56	61.91 ± 2.33
Uric acid level (mg.dL^−1^)	03.67 ± 1.34	03.41 ± 0.94
Bilirubin (mg.dL^−1^)	00.80 ± 0.87	00.90 ± 0.65
Urea (serum) level (mg.dL^−1^)	15.14 ± 2.01	15.88 ± 1.23
Creatinine (mg.dL^−1^)	01.19 ± 0.43	01.05 ± 0.74
Triglycerides level (mg.dL^−1^)	54.07 ± 2.03	53.71 ± 2.73
Alkaline phosphate (IU.L^−1^)	48.89 ± 1.99	52.86 ± 2.01
Aspartate transaminase (IU.L^−1^)	28.08 ± 2.13	27.39 ± 1.90
Alanine aminotransferase (IU.L^−1^)	143.46 ± 2.3	144.78 ± 2.1

Values are measured as mean ± SD (*n* = 3).

**Table 7:** Effects of administered of PVP-K30 nanogel formulation in the weights (g) of vital organs of test animals.

Animal groups	Heart	Liver	Lung	Kidney	Stomach	Spleen
Group C (control)	5.01 ± 0.43	6.99 ± 2.03	8.95 ± 1.67	13.05 ± 1.44	12.88 ± 1.39	1.85 ± 0.76
Group T (treated)	4.95 ± 0.37	7.21 ± 1.86	9.35 ± 2.00	12.92 ± 2.13	13.08 ± 2.04	1.93 ± 0.82

Values are measured as mean ± SD (*n* = 3).

## Data Availability

The data used to support the findings of this study are included within the article.

## References

[1] Ambrus R., Szabó-Révész P., Kiss T. (2020). Application of a suitable particle engineering technique by pulsed laser ablation in liquid (PLAL) to modify the physicochemical properties of poorly soluble drugs. *Journal of Drug Delivery Science and Technology*.

RETRACTED

[2] Jermain S. V., Brough C., Williams R. O. (2018). Amorphous solid dispersions and nanocrystal technologies for poorly water- soluble drug delivery - an update. *International Journal of Pharmaceutics*.

[3] Xie Y., Yao Y. (2018). Octenylsuccinate hydroxypropyl phytoglycogen, a dendrimer-like biopolymer, solubilizes poorly water-soluble active pharmaceutical ingredients. *Carbohydrate Polymers*.

[4] Bolourchian N., Nili M., Foroutan S. M., Mahboubi A., Nokhodchi A. (2020). The use of cooling and anti-solvent precipitation technique to tailor dissolution and physicochemical properties of meloxicam for better performance. *Journal of Drug Delivery Science and Technology*.

[5] Sharma M., Sharma R., Jain D. K., Saraf A. (2019). Enhancement of oral bioavailability of poorly water soluble carvedilol by chitosan nanoparticles: optimization and pharmacokinetic study. *International Journal of Biological Macromolecules*.

[6] Sanches B. M., Ferreira E. I. (2019). Is prodrug design an approach to increase water solubility?. *International Journal of Pharmaceutics*.

[7] Yousaf A. M., Ramzan M., Shahzad Y., Mahmood T., Jamshaid M. (2019). Fabrication andin vitrocharacterization of fenofibric acid-loaded hyaluronic acid–polyethylene glycol polymeric composites with enhanced drug solubility and dissolution rate. *International Journal of Polymeric Materials and Polymeric Biomaterials*.

[8] Bali N. R., Shinde M. P., Rathod S. B., Salve P. S. (2021). Enhanced transdermal permeation of rasagiline mesylate nanoparticles: design, optimization, and effect of binary combinations of solvent systems across biological membrane. *International Journal of Polymeric Materials and Polymeric Biomaterials*.

[9] Mao J., Wang H., Xie Y. (2020). Transdermal delivery of rapamycin with poor water-solubility by dissolving polymeric microneedles for anti-angiogenesis. *Journal of Materials Chemistry B*.

[10] Ghosal K., Adak S., Agatemor C., Praveen G., Kalarikkal N., Thomas S. (2020). Novel interpenetrating polymeric network based microbeads for delivery of poorly water soluble drug. *Journal of Polymer Research*.

[11] Naqvi A., Ahmad M., Minhas M. U., Khan K. U., Batool F., Rizwan A. (2020). Preparation and evaluation of pharmaceutical co-crystals for solubility enhancement of atorvastatin calcium. *Polymer Bulletin*.

[12] Veni D. K., Gupta N. V. (2020). Development and evaluation of Eudragit coated environmental sensitive solid lipid nanoparticles using central composite design module for enhancement of oral bioavailability of linagliptin. *International Journal of Polymeric Materials and Polymeric Biomaterials*.

RETRACTED

[13] Maheswari P. D., Rambhau D., Narasu M. L. (2020). Micelles entrapped microparticles technology: a novel approach to resolve dissolution and bioavailability problems of poorly water soluble drugs. *Journal of Microencapsulation*.

[14] Alam B. M., Aouak T., Alandis N. M., Alam M. M. (2015). Synthesis, characterization, drug solubility enhancement, and drug release study of poly (methacrylic acid-graft-simvastatin). *International Journal of Polymeric Materials and Polymeric Biomaterials*.

[15] Bi Y., Lv B., Li L. (2020). A liposomal formulation for improving solubility and oral bioavailability of nifedipine. *Molecules*.

[16] Alshweiat A., Csóka I. I., Tömösi F. (2020). Nasal delivery of nanosuspension-based mucoadhesive formulation with improved bioavailability of loratadine: preparation, characterization, and *in vivo* evaluation. *International Journal of Pharmaceutics*.

[17] Dong B., Hadinoto K. (2019). Carboxymethyl cellulose is a superior polyanion to dextran sulfate in stabilizing and enhancing the solubility of amorphous drug-polyelectrolyte nanoparticle complex. *International Journal of Biological Macromolecules*.

[18] Najafi F., Salami-Kalajahi M., Roghani-Mamaqani H., Kahaie-Khosrowshahi A. (2020). A comparative study on solubility improvement of tetracycline and dexamethasone by poly(propylene imine) and polyamidoamine dendrimers: an insight into cytotoxicity and cell proliferation. *Journal of Biomedical Materials Research Part A*.

[19] Potharaju S., Mutyam S. K., Liu M. (2020). Improving solubility and oral bioavailability of a novel antimalarial prodrug: comparing spray-dried dispersions with self-emulsifying drug delivery systems. *Pharmaceutical Development and Technology*.

[20] Siirilä J., Hietala S., Ekholm F. S., Tenhu H. (2020). Glucose and maltose surface functionalized thermoresponsive poly (N-vinylcaprolactam) nanogels. *Biomacromolecules*.

[21] Neamtu I., Rusu A. G., Diaconu A., Nita L. E., Chiriac A. P. (2017). Basic concepts and recent advances in nanogels as carriers for medical applications. *Drug Delivery*.

[22] Yadav H. K., Al Halabi N. A., Alsalloum G. A. (2017). Nanogels as novel drug delivery systems-a review. *Journal of Pharmacy and Pharmaceutical Research*.

[23] Navarro L., Theune L. E., Calderón M. (2020). Effect of crosslinking density on thermoresponsive nanogels: a study on the size control and the kinetics release of biomacromolecules. *European Polymer Journal*.

[24] Khan K. U., Minhas M. U., Badshah S. F., Suhail M., Ahmad A., Ijaz S. (2022). Overview of nanoparticulate strategies for solubility enhancement of poorly soluble drugs. *Life Sciences*.

RETRACTED

[25] Peltonen L. (2018). Practical guidelines for the characterization and quality control of pure drug nanoparticles and nano-cocrystals in the pharmaceutical industry. *Advanced Drug Delivery Reviews*.

[26] Zhang Y., Andrén O. C. J., Nordström R. (2019). Off-stoichiometric thiol-ene chemistry to dendritic nanogel therapeutics. *Advanced Functional Materials*.

[27] Kaur M., Sudhakar K., Mishra V. (2019). Fabrication and biomedical potential of nanogels: an overview. *International Journal of Polymeric Materials and Polymeric Biomaterials*.

[28] Richa A. R. C. (2020). Synthesis of a novel gellan-pullulan nanogel and its application in adsorption of cationic dye from aqueous medium. *Carbohydrate Polymers*.

[29] Suhail M., Rosenholm J. M., Minhas M. U. (2019). Nanogels as drug-delivery systems: a comprehensive overview. *Therapeutic Delivery*.

[30] Jain S., Ancheria R. K., Shrivastava S., Soni S. L., Sharma M. (2019). An overview of Nanogel–novel drug delivery system. *Asian Journal of Pharmaceutical Research and Development*.

[31] Zhuang T., Zhang W., Cao L. (2018). Isolation, identification and characterization of two novel process-related impurities in olanzapine. *Journal of Pharmaceutical and Biomedical Analysis*.

[32] Rudrangi S. R. S., Trivedi V., Mitchell J. C., Wicks S. R., Alexander B. D. (2015). Preparation of olanzapine and methyl-*β*-cyclodextrin complexes using a single- step, organic solvent-free supercritical fluid process: An approach to enhance the solubility and dissolution properties. *International Journal of Pharmaceutics*.

[33] Günther K. N., Banner J., Linnet K., Johansen S. S. (2020). Segmental hair analysis of olanzapine and *N*- desmethyl-olanzapine in postmortem hair from mentally ill patients by LC-MS/MS. *Journal of Pharmaceutical and Biomedical Analysis*.

[34] Jawahar N., Hingarh P. K., Arun R. (2018). Enhanced oral bioavailability of an antipsychotic drug through nanostructured lipid carriers. *International Journal of Biological Macromolecules*.

[35] Anup N., Thakkar S., Misra M. (2018). Formulation of olanzapine nanosuspension based orally disintegrating tablets (ODT); comparative evaluation of lyophilization and electrospraying process as solidification techniques. *Advanced Powder Technology*.

[36] Riman D., Rozsypal J., Halouzka V., Hrbac J., Jirovsky D. (2020). The use of micro carbon pencil lead electrode for sensitive HPLC-ED analysis of selected antipsychotic drugs. *Microchemical Journal*.

[37] de Freitas M. R., Rolim L. A., Soares M. F. L. R., Rolim-Neto P. J., Albuquerque M. M., Soares-Sobrinho J. L. (2012). Inclusion complex of methyl-*β*-cyclodextrin and olanzapine as potential drug delivery system for schizophrenia. *Carbohydrate Polymers*.

RETRACTED

[38] da Costa N. F., Fernandes A. I., Pinto J. F. (2020). Measurement of the amorphous fraction of olanzapine incorporated in a co- amorphous formulation. *International Journal of Pharmaceutics*.

[39] Zhang L., Hu Y., Jiang X., Yang C., Lu W., Yang Y. H. (2004). Camptothecin derivative-loaded poly(caprolactone-co-lactide)-b-PEG-b- poly(caprolactone-co-lactide) nanoparticles and their biodistribution in mice. *Journal of Controlled Release*.

[40] Shah S., Rangaraj N., Laxmikeshav K., Sampathi S. (2020). Nanogels as drug carriers - Introduction, chemical aspects, release mechanisms and potential applications. *International Journal of Pharmaceutics*.

[41] Khan K. U., Akhtar N., Minhas M. U. (2020). Poloxamer-407-co-poly (2-acrylamido-2-methylpropane sulfonic acid) cross-linked nanogels for solubility enhancement of olanzapine: synthesis, characterization, and toxicity evaluation. *AAPS PharmSciTech*.

[42] Khan K. U., Minhas M. U., Sohail M. (2021). Synthesis of PEG-4000-co-poly (AMPS) nanogels by cross-linking polymerization as highly responsive networks for enhancement in meloxicam solubility. *Drug Development and Industrial Pharmacy*.

[43] Khan K. U., Minhas M. U., Badshah S. F., Sohail M., Sarfraz R. M. (2022). *β*-cyclodextrin modification by cross-linking polymerization as highly porous nanomatrices for olanzapine solubility improvement; synthesis, characterization and bio-compatibility evaluation. *Journal of Drug Delivery Science and Technology*.

[44] Anwar M., Pervaiz F., Shoukat H. (2020). Formulation and evaluation of interpenetrating network of xanthan gum and polyvinylpyrrolidone as a hydrophilic matrix for controlled drug delivery system. *Polymer Bulletin*.

[45] Balamuralidhara V., Pramod Kumar T. M., Vishal Gupta N., Getyala A., Gangadharappa H. V. (2013). Development of a novel biodegradable superporous hydrogel for gastroretentive application. *International Journal of Polymeric Materials and Polymeric Biomaterials*.

[46] Jafar M., Khalid M. S., Aldossari M. F. E. (2020). Formulation of curcumin-*β* cyclodextrin–polyvinylpyrrolidone supramolecular inclusion complex: experimental, molecular docking and preclinical anti-nociceptive assessment. *Drug Development and Industrial Pharmacy*.

[47] Febriyenti P. I., Zaini E., Ismed F., Lucida H. (2020). Preparation and characterization of quercetin-polyvinylpyrrolidone K-30 spray dried solid dispersion. *Journal of Pharmacy & Pharmacognosy Research*.

[48] Asghar S., Akhtar N., Minhas M. U., Khan K. U. (2021). Bi-polymeric spongy matrices through cross-linking polymerization: synthesized and evaluated for solubility enhancement of acyclovir. *AAPS PharmSciTech*.

RETRACTED

[49] Tanveer S., Ahmad M., Minhas M. U., Ahmad A., Khan K. U. (2021). Chitosan-PVA-co-poly (2-acrylamido-2-methylpropane sulfonic acid) cross-linked hybrid IPN-nanogels for transdermal delivery of ondansetron; synthesis, characterization and toxicological evaluation. *Polymer-Plastics Technology and Materials*.

[50] Minhas M. U., Abdullah O., Sohail M. (2022). Synthesis of novel combinatorial drug delivery system (nCDDS) for co-delivery of 5-fluorouracil and Leucovorin calcium for colon targeting and controlled drug release. *Drug Development and Industrial Pharmacy*.

[51] Anandam S., Selvamuthukumar S. (2014). Fabrication of cyclodextrin nanosponges for quercetin delivery: physicochemical characterization, photostability, and antioxidant effects. *Journal of Materials Science*.

[52] Abbasi M., Sohail M., Minhas M. U. (2019). Novel biodegradable pH-sensitive hydrogels: an efficient controlled release system to manage ulcerative colitis. *International Journal of Biological Macromolecules*.

[53] World Health Organization (2009). WHO Expert Committee on Specifications for Pharmaceutical Preparations: Forty-third Report.

[54] Shah S. A., Sohail M., Minhas M. U. (2019). pH-responsive CAP-co-poly (methacrylic acid)-based hydrogel as an efficient platform for controlled gastrointestinal delivery: fabrication, characterization, in vitro and in vivo toxicity evaluation. *Drug Delivery and Translational Research*.

[55] Badshah S. F., Akhtar N., Minhas M. U. (2021). Porous and highly responsive cross-linked *β*-cyclodextrin based nanomatrices for improvement in drug dissolution and absorption. *Life Sciences*.

[56] Abuzar S. M., Hyun S. M., Kim J. H. (2018). Enhancing the solubility and bioavailability of poorly water-soluble drugs using supercritical antisolvent (SAS) process. *International Journal of Pharmaceutics*.

[57] Liu T., Yu X., Yin H. (2020). Study of top-down and bottom-up approaches by using Design of experiment (DoE) to produce meloxicam nanocrystal capsules. *AAPS PharmSciTech*.

[58] Christou C., Philippou K., Krasia-Christoforou T., Pashalidis I. (2019). Uranium adsorption by polyvinylpyrrolidone/chitosan blended nanofibers. *Carbohydrate Polymers*.

[59] Hancock B. C., Parks M. (2000). What is the true solubility advantage for amorphous pharmaceuticals?. *Pharmaceutical Research*.

[60] Long C. M., Tang K., Chokshi H., Fotaki N. (2019). Surface dissolution UV imaging for investigation of dissolution of poorly soluble drugs and their amorphous formulation. *AAPS PharmSciTech*.

RETRACTED

[61] Bode C., Kranz H., Fivez A., Siepmann F., Siepmann J. (2019). Often neglected: PLGA/PLA swelling orchestrates drug release: HME implants. *Journal of Controlled Release*.

[62] Wang W., Li M., Yang Q., Liu Q., Ye M., Yang G. (2020). The opposed effects of polyvinylpyrrolidone K30 on dissolution and precipitation for indomethacin supersaturating drug delivery systems. *AAPS PharmSciTech*.

[63] Taleb M. A., Hegazy D. E., Mahmoud G. A. (2014). Characterization and in vitro drug release behavior of (2-hydroxyethyl methacrylate)–co-(2-acrylamido-2-methyl-1-propanesulfonic acid) crosslinked hydrogels prepared by ionizing radiation. *International Journal of Polymeric Materials and Polymeric Biomaterials*.

[64] Hazer O., Soykan C., Kartal Ş. (2007). Synthesis and swelling behavior analysis of poly(acrylamidoxime‐co‐2‐acrylamido‐2‐methylpropane sulfonic acid) hydrogels. *Journal of Macromolecular Science, Part A: Pure and Applied Chemistry*.

[65] Wang W., Wang Q., Wang A. (2011). pH-responsive carboxymethylcellulose-g-poly (sodium acrylate)/polyvinylpyrrolidone semi-IPN hydrogels with enhanced responsive and swelling properties. *Macromolecular Research*.

[66] Yang J., Medronho B., Lindman B., Norgren M. (2020). Simple one pot preparation of chemical hydrogels from cellulose dissolved in cold LiOH/urea. *Polymers*.

[67] Yousaf A. M., Malik U. R., Shahzad Y., Mahmood T., Hussain T. (2019). Silymarin-laden PVP-PEG polymeric composite for enhanced aqueous solubility and dissolution rate: preparation and in vitro characterization. *Journal of pharmaceutical analysis*.

